The article "Recognition of Human Body Feature Changes in Sports Health Based on Deep Learning" was retracted in 2023. Reasons: unreliable results or conclusions; concerns about the data; concerns about the peer review; concerns about the citations.

# Recognition of Human Body Feature Changes in Sports Health Based on Deep Learning

**DOI:** 10.1155/2022/1736350

**Published:** 2022-03-24

**Authors:** Chendao Jiao

**Affiliations:** P.E. Scientific College, Harbin Normal University, Harbin, 150080 Heilongjiang, China

## Abstract

With the rapid development of social economy and the extensive and in-depth development of national fitness activities, national physical fitness monitoring and research work has achieved rapid development. In recent years, the application of deep learning technology has also achieved research breakthroughs in the field of computer vision. How deep learning technology can effectively capture motion information in sample data and use it to realize the recognition and classification of human actions is currently a research hot spot. Today's popularization of various shooting devices such as mobile phones and portable action cameras has contributed to the vigorous growth of image data. Therefore, through computer vision technology, image data is widely used in practical application scenarios of human feature recognition. This paper proposes a deep learning network based on the recognition of human body feature changes in sports, improves the recognition method, and compares the recognition accuracy with the original method. The experimental results of this paper show that the result of this paper is 1.68% higher than the original recognition method, the accuracy rate of the improved motion history image is increased by 14.8%, and the overall recognition rate is higher. It can be seen from the above experimental results that this method has achieved good results in human body action recognition.

## 1. Introduction

With the prosperity of sports, the demand for human body recognition technology has gradually increased. Human body feature recognition technology has a good auxiliary effect on activities in the sports field. Through the three-dimensional model, the human body's movement process can be better analyzed. At the same time, with the rapid development of mobile terminals, this technology has been widely used, which has also increased the growth of image data. Therefore, image data is widely used in actual scenes of human body feature recognition through computer vision. With the emergence of deep learning and the enhancement of computing power, deep learning and artificial intelligence methods are being used for automatic feature learning in different fields such as health and image classification. Recently, they are used for extraction and classification of simple and complex human activity recognition features in mobile devices. With the active development of sports in people's lives, the demand for human body feature recognition technology is increasing. The technology can help sports professionals perform 3D human modeling to analyze human movement in images.

The article "Recognition of Human Body Feature Changes in Sports Health Based on Deep Learning" was retracted in 2023. Reasons: unreliable results or conclusions; concerns about the data; concerns about the peer review; concerns about the citations.

At present, most of the research on human behavior recognition is focused on video data, which is based on the number of videos. At the same time, due to the complexity of video image data, it is easy to invade personal privacy. The recognition of human behavior characteristics has always been the focus of computer vision and artificial intelligence research. However, the behavioral characteristics of the human body not only contain spatial information but also need to further consider the dynamic characteristics of the human body. Therefore, the research on the extraction and classification of the human body's behavioral characteristics is very challenging.

The innovation of this article lies in two points. One is to recognize human body motion characteristics with the hot deep learning technology in recent years, and its own learning advantages can more accurately classify human body characteristics. The second is that this article has improved some of the recognition methods, and the experiment shows that the improved method has a better recognition effect than the unimproved method.

## 2. Relating Work

Deep learning algorithms have a wide range of applications and have played an important role in a variety of recognition and analysis fields. The prevalence of sports and health care has led many scholars to conduct in-depth research on the recognition technology of the human body in order to obtain better auxiliary effects. The continuous development of science and technology puts forward higher requirements for sports research. Hou analyzed the topic description and behavior recognition based on human motion visual features, mainly introduced the main content of feature extraction and description, and discussed the main content and research methods of human behavior recognition in the thesis. The results show that the improved algorithm proposed has a good effect on behavior recognition and provides a new idea for future research on feature extraction and recognition of sports behavior [1]. Shin and Cha propose a new system to overcome the problems existing in the two existing methods of identifying diverse and complex human behaviors. These two methods are the direct sensor measurement method and the artificial intelligence-based method. In order to realize this system, a multimodal sensor composed of acceleration, gyroscope, and height sensors was developed, and a method that combines sensor measurements and deep learning research results in real time to more accurately recognize gestures and behaviors is described. The practicability and effectiveness of the proposed system are verified by experiments in a real environment [2]. The main purpose of various methods of evaluating athletes' feature recognition is to monitor the athlete's current health status, so as to provide some feedback on the quality of individual training. Based on deep learning and convolutional neural network, Liu and Ji study the target recognition of athletes and propose a feature vector extraction method based on the zero point of curvature. In addition, on the basis of their ideas, they constructed an athlete feature recognition model and optimized the algorithm. The research results show that the proposed method has certain advantages in athlete feature extraction and can be used in subsequent sports training systems [3]. Because the existing player evaluation methods rely heavily on game statistics, they cannot capture the qualitative impact of each player in the game. By combining quantitative game statistics and qualitative analysis provided by news articles, Park et al. propose a player evaluation model in deep learning-based approach. The proposed system was applied to the Korean Professional Baseball League (KBO), and it was proven to be able to understand the sentence polarity of news articles about player performance [4]. Under the influence of COVID-19, there is a great need for research on behavior recognition. Zheng et al. proposed a recurrent neural network algorithm based on long- and short-term memory (LSTM) to realize the recognition of behavior patterns, thereby improving the accuracy of human activity behavior recognition [5]. Improving the level of sports has always been a concern of my country's sports industry. With the continuous improvement of the computer level, how to effectively identify the trajectory of the movement has become a hot spot in the research of related institutions. Based on this, Baoshan researched a motion recognition method based on depth information. First, it briefly introduces the basic knowledge of related theories, including general methods of motion recognition, and the use of depth information for motion recognition. On this basis, a motion recognition method based on depth information is proposed [6]. The above-mentioned scholars have high demand for related research, all require a solid theoretical foundation and are not easy to operate. And it is not easy to collect complete and comprehensive information in data collection.

The article "Recognition of Human Body Feature Changes in Sports Health Based on Deep Learning" was retracted in 2023. Reasons: unreliable results or conclusions; concerns about the data; concerns about the peer review; concerns about the citations.

## 3. Human Feature Recognition Based on Deep Learning

### 3.1. Human Body Recognition Based on Deep Learning

#### 3.1.1. The Nature of the Depth Image

In 3D computer graphics, a depth map is a special image, which is different from the traditional gray-scale image where the pixel points represent the pixel intensity value. The depth image records the distance information from the camera to the surface of the scene object [7]. The reason why the depth image is also called the distance image is because the change of the pixel value in the depth map corresponds to the change of the distance in the real three-dimensional world, and the real three-dimensional scene can be reflected by the difference in the depth value [8, 9]. In the human action recognition based on the depth image, each pixel (x, y) in the depth image represents the distance of each part of the human body from the depth camera plane [10]. Normally, RGB image and depth image are obtained at the same time, so their pixels are in a completely contrasting relationship. Due to the unique properties of depth images, depth images are often not disturbed by complex backgrounds, and there is no need to design foreground extraction algorithms for them. Only using the distance information in the depth map to obtain foreground target information requires feature extraction to make the entire recognition system relatively simple.

According to the above description, two properties of depth images are obtained: Color independence and changes in pixel values correspond to changes in the *Z* axis of the three-dimensional world [11]. Color independence means that the depth image is not sensitive to environmental factors such as the surface color, shadow, and lighting of the object. Another feature of the depth map can be used to separate the various parts of the same object, which causes the problem of overlapping parts of the same object solved in a certain sense. And the use of depth images can be used to reconstruct a part of an object in three dimensions [12].

#### 3.1.2. Commonly Used Human Motion Recognition Database

In view of the fact that most of the current work is mostly tested and verified in the public video database, therefore, the collection of the database plays a vital role in the recognition of human actions. Nowadays, more and more human movement databases are made public. The early databases were all RGB color image databases, and the most widely used ones were Weizmann and KTH [13]. The actions in these two databases are relatively simple, the background is relatively simple and static, and the fixed angle of view is used when recording, so the difficulty of identification is relatively low. In recent years, some databases with complex backgrounds, rich types of actions, and interactive actions have appeared one after another, for example, Hollywood2 database, UCF sports database, UCF101 database, and HMDB51 database [14]. In addition, the IXMAS database is mainly used for human action recognition in multiview scenes.

The article "Recognition of Human Body Feature Changes in Sports Health Based on Deep Learning" was retracted in 2023. Reasons: unreliable results or conclusions; concerns about the data; concerns about the peer review; concerns about the citations.

### 3.2. Action Feature Extraction

In the field of computer vision, if the computer is to be able to understand the image, to realize the real “vision.” This requires extracting useful data or information from the image and expressing it in a digitized form (such as numerical values or vectors). This process is feature extraction [15].These extracted digital representations are features. Then, through the training of these features, the computer has the ability to recognize images [16].

#### 3.2.1. Depth Motion Maps

Depth Motion Map (DMM) is a projection map model designed specifically for depth images. It first projects each frame of the action video sequence onto three orthogonal Cartesian planes (xoy plane, xoz plane, and yoz plane). In this way, each frame of the depth image of the entire sequence can be viewed from the front view (mapf), the side view (maps), and the top view (mapt). After removing the areas where there is no human body motion on each projection image, the projection image is normalized by bilinear interpolation to reduce the interference caused by the difference of personal height and range of motion [17]. Then, calculate the absolute value difference between two consecutive frames before and after each view, and the difference between the absolute value difference and a certain set threshold is called the motion energy. Movement energy reflects where the action occurs during the duration of the action and provides important discriminant information for identifying the type of action. Then, the motion energy of the entire sequence is accumulated to obtain the depth motion map of the action sequence [18]. The calculation formula of the depth motion map (DMMv) in each view is as follows:

(1) $$\begin{array}{c} \text{BWW}\wedge =\overset{\text{d}}{\underset{t=d}{\sum }}\left(\left|{MAP}_{\wedge }^{t+1}-{MAP}_{\wedge }^{t}\right|>\alpha \right). \end{array}$$

In the above equation, ∧∈{y, *h*, *i*}, and *y*, *h*, and *i*, respectively, represent the three perspectives of front, side, and top, and *d* is the label of the end frame. The projection of the action of the *t*th frame under the view angle ∧ is MAP_∧_^t^. *α* is the manually input threshold.

#### 3.2.2. Histograms of Oriented Gradients

The HOG descriptor was first proposed by French researcher Dalal at the CVPR2005 conference and has achieved good results in pedestrian detection [19]. HOG can be applied to the feature extraction of RGB images and depth images. Because the edge of the image is the region with the most gradient distribution, the gradient direction histogram can well describe the shape and appearance information of the object. It calculates the weighted projection of the gradient magnitude in the gradient direction in some regions of an image and then connects each local region to form the final feature. Its calculation steps are as follows:

1. Normalized image: since the changes in illumination and shadow have a greater impact on the texture intensity of the image, in order to reduce the influence of these factors, the commonly used method is to normalize the image [20]. Here, the image is grayed out first, and then, Gamma compression is used for the gray image obtained
2. The calculation equation of the gradient size *W* (*A*, *B*) and direction *S* (*A*, *B*) of the pixel is

(2) $$\begin{array}{c} W\left(A,B\right)=\sqrt{{\left[q\left(A+1,B\right)-q\left(A-1,B\right)\right]}^{2}+{\left[q\left(A,B+1\right)-\left(A,B-1\right)\right]}^{2}}, \end{array}$$

(3) $$\begin{array}{c} S\left(A,B\right)=arc\frac{q\left(A+1,B\right)-q\left(A-1,B\right)}{q\left(A,B+1\right)-q\left(A,B-1\right)}, \end{array}$$

where *W* (*A*, *B*) is the gradient amplitude value of a certain pixel, *S* (*A*, *B*) represents the direction of the gradient, and *q* (*A*, *B*) represents the pixel value of a certain point

(3) Constructing the histogram of the gradient direction of the image: first, dividing an image into grids. These grids are called cells. Dividing the 360-degree circle into a number of artificially set bins and then calculating the histogram of the weighted projection of each pixel of the image in these small areas according to the gradient direction. Finally, connecting the histograms of these cell units in series, and then using L2-norm to normalize the entire gradient histogram to further reduce the interference of external environmental factors. Finally, the normalized histogram is the final feature descriptor. The L2-norm calculation formula is as follows:

(4) $$\begin{array}{c} \wedge ⟶\vee /\sqrt{{\left\|\left(\vee \right)\right\|}_{2}^{2}+\alpha } \end{array}$$

The article "Recognition of Human Body Feature Changes in Sports Health Based on Deep Learning" was retracted in 2023. Reasons: unreliable results or conclusions; concerns about the data; concerns about the peer review; concerns about the citations.

#### 3.2.3. Local Binary Patterns

Local Binary Pattern (LBP) is often used to describe the local texture information of an image in the field of computer vision and pattern recognition. Because the texture information described has a high degree of discrimination, it is fast and convenient to implement, has a small amount of data, and has gray-level invariance and rotation invariance. In the early days, it was mostly used in research directions such as target detection and face recognition. The LBP compares the gray value of the central pixel with the relationship between the gray value of other pixels in the space and then encodes this relationship to achieve the purpose of describing texture features [21].

The most basic LBP descriptor is a 3 × 3 neighborhood structure, as shown in Figure 1. In the figure, 139 is the LBP value of the central pixel in this square area. However, this square field can only encode a fixed range and cannot adapt to changes in image scale. Subsequently, some scholars proposed a circular field to solve this problem, which can calculate the LBP value of any number of pixels in different radius ranges.

Assuming that Q*a*(*A*0, *B*0) is the center of the pixel, then, there are *w* domain points uniformly distributed on the radius *R* of the circle. The coordinates are as follows:

(5) $$\begin{array}{c} \left(\text{A}0-R\sin\left(2\pi t/w,B0+\cos\left(2\pi t/w\right)\right)\right). \end{array}$$

Since sampling is performed on a circle, the coordinate values of some points may not be integers. But the pixel value of the image must be an integer, so the bisexual interpolation method is mostly used to estimate the value of the coordinate. The calculation equation of the LBP of Q*a* under the circular field framework is as follows:

(6) $$\begin{array}{c} \text{LBP}\left(w,R\right)\left(Qa\right)=F\left(y\left(Bt\right)\right), \end{array}$$

(7) $$\begin{array}{c} Bt=Qt-Qa, \end{array}$$

(8) $$\begin{array}{c} F\left(m\right)=\overset{m‐1}{\underset{t=0}{\sum }}mt\cdot 2^{t}, \end{array}$$

(9) $$\begin{array}{c} y\left(Qa\right)=\left\{\begin{array}{cc} 1 & Qa\geq 0\\ 0 & Qa<0 \end{array}\right.. \end{array}$$

In the above equation, *F*(*m*) represents a function that can convert the *x*-bit binary to the decimal system, and the difference from the *t*th point to the center pixel is *Bt*. As shown in Figure 2, the radius *R* = 1, and the number of fields is 8.

### 3.3. Action Classification Recognition

After feature extraction, a feature vector that can effectively describe human actions is obtained. In general, the dimensionality of the feature vector is relatively high and contains more redundant information. If it is directly sent to the classifier, not only will the calculation amount be quite large, but some invalid information may affect the accuracy of recognition. Therefore, it is necessary to reduce the dimensionality of the original feature vector. While avoiding the disaster of dimensionality, it also obtains the most important component of the feature vector and saves memory at the same time. At present, the commonly used dimensionality reduction methods mainly include linear dimensionality reduction (PCA) and nonlinear dimensionality reduction (manifold learning and local linear embedding). In this paper, principal component analysis (PCA), which is relatively simple in calculation, is mainly used for feature dimensionality reduction [22].

The article "Recognition of Human Body Feature Changes in Sports Health Based on Deep Learning" was retracted in 2023. Reasons: unreliable results or conclusions; concerns about the data; concerns about the peer review; concerns about the citations.

In addition, some classifiers based on probability graph models are often used to identify classification problems. They mainly calculate the conditional probabilities of the data to be classified (observed data) under all labels. Under which label has the highest probability, it means that the current data belongs to the category represented by this label. The most representative ones are Bayesian networks and random field models [23]. There are also some commonly used classifiers, such as random forest, AdaBoost classifier, and artificial neural network, which are widely used in various fields [24]. The following is a detailed introduction to the classifier used in this article.

### 3.4. Support Vector Machine.

#### 3.4.1. SVM Is Linearly Separable

There are two types of data on the two-dimensional plane as shown in Figure 3, which are represented by circles and squares. For these linearly separable data, you only need to find a cutting line that can perfectly separate the two types of data [25].

While maximizing the classification interval, it is necessary to ensure that the classification of other sample points is correct. The constraints are as follows:

(10) $$\begin{array}{c} Bt\left(m^{i}A+d\right)\geq 1. \end{array}$$

So this classification problem is transformed into a problem of minimizing the following objective function under the above constraints.

(11) $$\begin{array}{c} \beta \left(m\right)=\frac{1}{2}m^{i}m. \end{array}$$

The constructed Lagrange function is

(12) $$\begin{array}{c} \text{La}\left(m,d,\chi \right)=\frac{1}{2}m^{i}m-\overset{n}{\underset{t=1}{\sum }}\chi \left[Bt\left(m^{i}At+d\right)-1\right]. \end{array}$$

Solving Equation (12), the optimal solution *χ*^∗^, *m*^∗^, and *d*^∗^ of *χ*, *m*, and *d* is obtained, so the optimal classification function can be expressed as

(13) $$\begin{array}{c} H\left(b\right)=\mathrm{sgn}\left(m^{*}b+d^{*}\right)=\mathrm{sgn}\left[\overset{n}{\underset{t=1}{\sum }}\chi^{*}At\left(bt\cdot b\right)+d^{*}\right]. \end{array}$$

#### 3.4.2. SVM Is Inseparable Linearly

In the case of linear inseparability, SVM solves this problem by introducing a kernel function, which plays a crucial role in the classification of SVM, it does not carry out the calculation of the data in the high-dimensional space after the kernel function is mapped, and the main calculation amount still occurs in the low-dimensional space. Here, the kernel function only plays the role of a space transformation and dimensional space to calculate the optimal hyperplane. But it is often difficult to construct a new kernel function. So the simplest method is to directly select and use from the existing kernel functions [26]. The three commonly used kernel functions are as follows:

Polynomial:

(14) $$\begin{array}{c} {\left(A^{t}At+1\right)}^{q}, \end{array}$$

where *q* represents the power parameter.

The article "Recognition of Human Body Feature Changes in Sports Health Based on Deep Learning" was retracted in 2023. Reasons: unreliable results or conclusions; concerns about the data; concerns about the peer review; concerns about the citations.

Hyperbolic tangent:

(15) $$\begin{array}{c} \tan\left[\delta 0A^{t}At+\delta 1\right], \end{array}$$

where *δ*0 and *δ*1 both represent specially selected parameters.

RBF is

(16) $$\begin{array}{c} \text{ex}\left[-\frac{1}{2\theta^{2}}{\left\|A-At\right\|}^{2}\right], \end{array}$$

where *θ*^2^ is an optional parameter.

For linear and inseparable problems, you need to map the data to a high-dimensional space.

(17) $$\begin{array}{c} A⟶{\left\{\left(\varphi \left(\text{At}\right)\right.\right\}}_{t=1}^{w1}. \end{array}$$

The classification hyperplane constructed in high-dimensional space is

(18) $$\begin{array}{c} \overset{n}{\underset{t=1}{\sum }}\chi tBt\varphi \left(At\right)\varphi \left(A\right)=0. \end{array}$$

At this time, the defined kernel product is

(19) $$\begin{array}{c} R\left(A,At\right)=\varphi^{t}\left(A\right)\varphi \left(At\right)=\overset{n}{\underset{t=1}{\sum }}\varphi t\left(A\right)\varphi t\left(At\right). \end{array}$$

Based on the same idea of linear separability, the problem is transformed into:

(20) $$\begin{array}{c} \max\overset{n}{\underset{t=1}{\sum }}\chi t-\frac{1}{2}\overset{n}{\underset{t=1}{\sum }}\overset{n}{\underset{t=1}{\sum }}\chi t\chi BtR\left(A,At\right), \end{array}$$

(21) $$\begin{array}{c} \overset{n}{\underset{t=1}{\sum }}\chi tBt=0,\;0\leq \chi t\leq D. \end{array}$$

In Equation (21), *D* is a positive parameter selected by the user, and Equation (21) is a constraint condition. After the equation is constructed and solved, the parameters are substituted into Equation (18) to obtain the optimal decision surface.

### 3.5. Challenges Faced by Human Feature Recognition

Human action recognition has been developed rapidly in the last ten years. In order to make action recognition can be well applied in real life, more and more effective and robust methods have been proposed. These methods are often more inclined to be applied in real life scenarios. Although relatively ideal recognition results have been achieved, there are still many thorny problems and challenges.

#### 3.5.1. Interference from the External Environment

The interference of the complex external environment has always been a big problem in the field of action recognition. Complicated backgrounds, including messy backgrounds, dramatic changes in illumination, and camera shake, make it extremely difficult to extract the foreground. Occlusion generally occurs in relatively complex interactive actions. For example, in multiperson interactive actions, the occlusion of actions between people makes the recognition of the overall interactive actions inaccurate. In addition, in the case of camera movement, the expression of human actions in different viewing angles is very different, so it is also a great challenge to extract robust features for recognition in a multiview environment.

The article "Recognition of Human Body Feature Changes in Sports Health Based on Deep Learning" was retracted in 2023. Reasons: unreliable results or conclusions; concerns about the data; concerns about the peer review; concerns about the citations.

#### 3.5.2. It Is Difficult to Recognize Continuous Unsegmented Actions and Complex Actions

Since human body movements are a continuous process in time, there is no clear sign to indicate the end of the previous movement and the beginning of the next movement, which makes it often difficult to distinguish a single movement. At this stage, most of the data used in the research is segmented and marked action data. Good results have been achieved in the recognition of relatively simple single actions, simple interactions between two people, and interactions between a single person and a single object. However, the recognition effect for those continuous undivided actions, complex multiperson interaction actions, and group behaviors is not ideal.

#### 3.5.3. The Influence on Recognition within and between Action Types

For the same action, different people will behave differently when performing the action, which results in different amplitude and duration of the same action. In this way, in the design of the feature extraction method, the spatial scale and movement speed should not be deformed. In addition, there may also be greater similarities between different actions, which brings great difficulties to the accurate recognition of actions. For example, “Draw a cross” and “Draw a circle” have a very high similarity, resulting in a high rate of misjudgment of the recognition results.

## 4. Convolutional Neural Network

In recent years, deep neural networks have gradually become a very popular research direction and have made breakthroughs in computer vision and other fields. Accurately detecting and extracting key regions of human motion from video is the first step in human action recognition, and its accuracy will directly affect the effect of subsequent action recognition tasks. The deep convolutional neural network is greatly affected by the dataset in the training stage, and the size of the samples in the dataset directly affects the structure and performance of the network. As an important branch of deep neural networks, convolutional neural networks are widely used in video image, speech recognition, and other fields. Its appearance also provides a new solution for the human action recognition problem that we are studying.

The article "Recognition of Human Body Feature Changes in Sports Health Based on Deep Learning" was retracted in 2023. Reasons: unreliable results or conclusions; concerns about the data; concerns about the peer review; concerns about the citations.

### 4.1. Common Convolutional Network

Convolutional neural networks are mostly used for image classification, detection, and recognition tasks. Structurally, in a convolutional neural network, the convolutional layer and the subsampling layer can form a feature extractor. In the convolutional layer, a mechanism called “local receptive field” is used, which means that neurons are not connected to all neurons in the adjacent layer, but are partially connected. Second, another feature of the network is shared weights. The so-called shared weights refer to the use of convolution kernels of the same size. In addition, subsampling is also a major feature. Subsampling is also called pooling, and there are two methods commonly used: mean pooling and maximum pooling. Mean pooling means that the center point coordinates take the average value of the elements covered by the pooled template, and maximum pooling means that the maximum value of the elements is taken. The different combinations of these features or mechanisms have become the cornerstones of some of our commonly used convolutional neural network structures today. Its advantage is that it can greatly reduce the number of weights and greatly reduce the complexity of the model. The main convolutional neural networks involved in this article are AlexNet and GoogleNet. Then, I will introduce these two networks.

#### 4.1.1. AlexNet

AlexNet was published in 2012 and became an instant hit. It can be called a classic of the year [27]. The emergence of AlexNet has reversed the decline of convolutional neural networks and inspired the confidence of scholars in this field. Many more excellent networks have been proposed one after another. When participating in the ImageNet competition that year, the top5 error rate was only 19.8%. Compared with the previous machine learning classification algorithm, the network is already very impressive. The model is divided into eight layers in total, including five convolutional layers and three fully connected layers, and each convolutional layer contains a linear rectification function and a local response normalization process and then undergoes a pooling process. The specific structure distribution is shown in Figure 4.

In general, pooling is nonoverlapping, while the pooling used by AlexNet is overlapping, that is, when pooling, the step length of each move is smaller than the side length of pooling. After the pooling is completed, the network sets up a local corresponding normalization mechanism, which can increase the generalization ability, smoothly process the data, and improve the recognition rate. The calculation formula is shown in formula (22).

(22) $$\begin{array}{c} d_{a,b}^{t}=\frac{\alpha_{a,b}^{t}}{\left(R+\alpha \sum_{t=\max\left(0,t-1\right)}^{\min\left(n-1,t+n/2\right)}{\left(\alpha_{a,b}^{t}\right)}^{2}\right)}. \end{array}$$

The equation shows that multiple values before and after a value are standardized, where the value of the *t*th convolution (*a*, *b*) coordinate is expressed as *α*_a,*b*_^*t*^, and *R*, *n*, and *α* are all hyperparameters.

The article "Recognition of Human Body Feature Changes in Sports Health Based on Deep Learning" was retracted in 2023. Reasons: unreliable results or conclusions; concerns about the data; concerns about the peer review; concerns about the citations.

#### 4.1.2. GoogleNet

One common point of the two models, GoogleNet and VGG, is that there are more layers and a deeper network structure. Structurally speaking, VGG inherits some frameworks of Lenet and alexNet. Unlike VGG, GoogleNet has made a bolder attempt on the Internet. Although this model has 22 layers, its size is much smaller than AlexNet and VGG, and it still performs well [28]. The most effective way to obtain a higher-quality model is to increase the number of layers (that is, depth) of the model or the number of convolution kernels or neurons in each layer of the model (model width).

The GoogleNet model has 22 layers, and the number of layers is deeper. At the same time, in order to avoid the gradient dispersion problem mentioned earlier, GoogleNet cleverly added two loss functions at different depths to eliminate the gradient dispersion phenomenon. Not only has the network depth increased, GoogleNet has also increased the network width, thereby reducing the complexity of the feature map and achieving the effect of dimensionality reduction, as shown in Figure 5. In addition, the use of this modular structure design can also facilitate the addition and modification of the network structure.

In addition, GoogleNet has made the following improvements:

1. The network finally uses average pooling to replace the fully connected layer. This idea originates from NIN, the reason why NIN uses a multilayer perceptron is that the structure of MLP is compatible with CNN, both can be trained using backpropagation, and it is also a deep model, which is consistent with the concept of feature reuse. And experiments have shown that this method can increase the accuracy of TOP-1 by 0.6%
2. In order to solve the problem of gradient disappearance caused by the deepening of the network layer, the network designed two branches and added two softmax classifiers at the end of the branches to assist in adjusting the network parameters. Some researchers have proposed to add attenuation coefficients to the two classifiers, but in the end, it is proved through experiments that the improvement is not very meaningful [29, 30]. When we actually test, these two extra softmax will be removed, only based on the output result of the main softmax. Softmax maps some inputs to real numbers between 0 and 1, and the normalization guarantees that the sum is 1, so the sum of the probabilities of multiclassification is exactly 1. It is widely used in multiclassification scenarios

The article "Recognition of Human Body Feature Changes in Sports Health Based on Deep Learning" was retracted in 2023. Reasons: unreliable results or conclusions; concerns about the data; concerns about the peer review; concerns about the citations.

### 4.2. Recognition Based on Deep Learning Network

#### 4.2.1. Result Analysis

In order to compare the performance of the two networks AlexNet and GoogleNet in this article, the experiment uses the color motion history image and the front view of the depth motion map as data, trains the network from zero under the same conditions, and compares and analyzes the experimental performance of the two networks.

From the data in Figure 6, we can find that, not in all data, the deeper the network and the more layers, the higher the recognition accuracy. When the input data is motion history images, AlexNet outperforms GoogleNet, with a recognition accuracy of 75% and 72%, respectively, and the latter has a deeper and wider network structure. When the input data is a front view, the recognition accuracy of the two is 74% and 76%, respectively, and the effect of GoogleNet is relatively good. Therefore, we can conclude that when the amount of training data is small, the recognition effect of the network with fewer layers is better, and the network with a deeper structure is slightly less effective. This is because the deep structure network has more parameters that need to be optimized and adjusted, and a small amount of data cannot train the parameters well.

#### 4.2.2. Fine-Tuning the Network

Due to insufficient data volume, the parameters cannot be adjusted optimally. At this point, if there is a model with pretrained parameters, we adjust it on the basis of it to adapt it to the problem we want to solve; then, things become less tricky. This process is called fine-tuning. In this article, we choose the AlexNet and GoogleNet networks trained on the ImageNet dataset. ImageNet is an image dataset organized according to the WordNet hierarchy and is free for academic research and noncommercial use. First, we need to download the trained caffemodel. Then, the entire process of network fine-tuning is shown in Figure 7.

### 4.3. Drawing of Precision Curve and Loss Function Curve

In the Caffe training process, in order to better understand the convergence of the network and show your own results, you usually graph your own training data. This not only facilitates the adjustment of parameters during the training process but also facilitates the display of the final results. The graph finally obtained is shown in Figure 8.

Figure 8(b) is a graph of the test accuracy and the number of iterations. After the increase, the overall trend is stable within a range. Figure 8(a) is a graph of the loss function and the number of iterations. At the beginning of the iteration, it shows a sudden downward trend and then tends to a stable state.

The article "Recognition of Human Body Feature Changes in Sports Health Based on Deep Learning" was retracted in 2023. Reasons: unreliable results or conclusions; concerns about the data; concerns about the peer review; concerns about the citations.

## 5. Human Body Characteristics Based on Deep Learning

### 5.1. Two Deep Learning Networks Experimental Results

Because these two types of data have orders of magnitude difference. As shown in Table 1, the amount of training data and test data of the exercise history graph and the side view and top view data amount of the experiment in this article are also listed in the table. The training network structure still uses two deep learning networks, AlexNet and GoogleNet, and the training starts from the most primitive state. The experimental results are shown in Figures 9(a) and 9(b).

It can be seen from the experimental results that whether it is the motion history image as the input or the front view of the depth motion map as the input, and whether it is AlexNet or GoogleNet in the network framework, Fine-tuning on the trained model has a higher recognition accuracy than restarting the training. At the same time, it can also be found that the recognition accuracy obtained by fine-tuning the motion history image on AlexNet is higher than that on GoogleNet, while the situation of the depth motion image is just the opposite. This is why this article finally chose to fine-tune AlexNet for motion history images and fine-tune GoogleNet for deep motion images.

### 5.2. Feature-Level Fusion and Decision-Level Fusion

Information fusion, also known as data fusion, refers to the integration of different information together to remove redundancy. The information obtained after fusion will benefit our subsequent analysis and processing. In the field of image processing, information fusion is divided into three types: data fusion, feature fusion, and decision fusion. The fusion of data or sample level in the data acquisition and preprocessing stages is called data fusion, the combination of features in the feature extraction stage is called feature fusion, and the fusion of recognition results in the classification decision stage is called decision fusion. This article uses feature fusion and decision fusion, so the following two parts of the content are related experiments and explanations.

#### 5.2.1. Feature Level Fusion

This article is mainly based on the convolutional neural network to extract features, then performs feature splicing, and then uses the softmax classifier to train and classify the spliced features. The overall framework is shown in Figure 10.

The result is shown in Figure 11. From the table, we can see that the more feature samples and the higher the feature dimension, the better the classification effect of the trained classifier. When we stitch all the four features, the classification effect is the best.

The article "Recognition of Human Body Feature Changes in Sports Health Based on Deep Learning" was retracted in 2023. Reasons: unreliable results or conclusions; concerns about the data; concerns about the peer review; concerns about the citations.

#### 5.2.2. Decision-Level Integration

Decision fusion refers to the training of multiple features to obtain multiple classifiers, and then, these classifiers are combined according to different rules, and finally a target judgment result is obtained under the common action. In this article, the front view, side view, and top view of the motion history image and the depth motion map are mainly used to train the convolutional neural network to obtain four classification results. Then, we use different rules to fuse these four classifiers, as shown in Figure 12.

### 5.3. Recognition of Different Fusion Rules Based on Deep Learning

This article uses the five different fusion rules listed in the table to conduct experiments.

It is not difficult to find from Table 2 that by using different fusion rules to combine the recognition results of the motion history map, the front view of the depth motion map, the side view, the top view, and different final recognition accuracy rates can be obtained. Among them, the results of the four kinds of motion characterization images are fused by the multiplication rule, and the highest recognition accuracy can be obtained in the end.

### 5.4. Recognition Accuracy of Different Verification Methods Based on Deep Learning

This section first conducts experiments on different verification methods and different decision fusion methods and compares their accuracy. The experimental results are shown in Table 3. It can be seen from the table that there will be big differences in the effects of different performers of the same type of action, and the same actions will also show differences. Because even if the same target verification is used, the recognition accuracy cannot reach 100%. But in comparison, same-target verification is more accurate than cross-target verification. But at the same time, cross-target verification can better explain the robust performance and generalization performance of the trained model.

As shown in Figure 13, we have done the same experiment for comparison. The results prove that the improvements made in this article on the motion history image and the depth motion map and the selection of a more appropriate network for different numbers of networks have an effect on the accuracy of recognition. The depth motion map uses the average rule for decision fusion, and the result of this paper is 1.68% higher than the original recognition method. The improved motion history image accuracy rate has increased by 14.8%, and when the depth motion map and the motion history map are fused by the average rule, it is increased by 2.4%, and when the multiplication rule is used, it is increased by 0.69%.

The article "Recognition of Human Body Feature Changes in Sports Health Based on Deep Learning" was retracted in 2023. Reasons: unreliable results or conclusions; concerns about the data; concerns about the peer review; concerns about the citations.

Figure 14 shows the comparison of the recognition rate of each type of action between the method in this paper and the unimproved method. It can be seen that there are 17 categories where the action recognition rate reaches 100% in this paper, while only 13 categories have not improved methods. Although the recognition rate of some actions is not as high as that of the unimproved method, the overall recognition rate is higher. It can be seen from the experimental results that this method has achieved good results in human action recognition. At the same time, the RGB video and depth video captured by the depth camera are used, and the motion history map and the depth motion map are used to represent and enhance the motion information. Combined with the convolutional neural network, four parallel network architectures are used, which can combine depth information with RGB video information and improve the accuracy of action recognition.

## 6. Conclusions

This article briefly introduces the convolutional neural network and the internal structure of the two networks selected in this article. Then, three methods of information fusion are introduced, and two fusion methods experimented in this paper are described in detail. Finally, at the end of this chapter, the experiments done at this stage and the analysis of their results are given. This paper mainly studies the recognition and classification of human actions combined with deep learning. First of all, human action contains time dimension information and spatial dimension information in the execution process, which is of great significance to the recognition of the action. How to extract and characterize the movement information is particularly important. Secondly, how to effectively use the characterization information for action recognition and classification also has a great influence on the final result. Finally, for small-scale databases, how to make full use of limited data to achieve higher accuracy is also a problem that needs to be solved. In response to the above problems, this paper has conducted some related studies. The results show that the same-target verification is more accurate than cross-target verification, but at the same time, cross-target verification can better explain the robust performance and generalization performance of the trained model. The comparison of the action recognition rate between the method in this paper and the unimproved method shows that the improved method is more excellent.

The article "Recognition of Human Body Feature Changes in Sports Health Based on Deep Learning" was retracted in 2023. Reasons: unreliable results or conclusions; concerns about the data; concerns about the peer review; concerns about the citations.

## Figures and Tables

**Figure 1:** The calculation process of the LBP value of the central pixel in the square area.

**Figure 2:** Schematic diagram of the LBP of a circular field with 8 fields.

**Figure 3:** Linear separability diagram of support vector.

**Figure 4:** The first layer network structure of AlexNet.

**Figure 5:** Inception module of GoogleNet network.

**Figure 6:** The recognition accuracy of different networks when the input values are different.

**Figure 7:** Basic steps for fine-tuning the network.

**Figure 8:** Test curve of exercise history graph.

**Figure 9:** Comparison of the recognition rate of the two networks under the two methods of training and fine-tuning.

**Figure 10:** Schematic diagram of feature stitching.

**Figure 11:** Recognition rate of different stitching features.

**Figure 12:** Flow chart of decision fusion.

**Figure 13:** Comparison of the recognition effect of the original and the improved recognition effect of different methods.

**Figure 14:** The recognition rate of each type of action of the method in this paper and the unimproved method.

**Table 1:** Number of training data and test data.

	MHI	Front	Side	Top
Training samples	435	3798	3798	3798
Test data	429	429	429	429
Mean	432	2113.5	2113.5	2113.5

**Table 2:** Accuracy of recognition under different fusion rules.

Law of fusion	Recognition rate%
3331Mfst	87.5
Fst	89.6
442fst	89.6
Mfst(+)	91
Mfst(∗)	91.8

**Table 3:** Recognition accuracy under different verification methods.

Ways of identifying Fusion decision	Multiplication rule	Law of peace	Weight rule
Same target verification	99.5	98.1	98.8
Cross-target verification	91.9	91.8	87.6
Mean	95.7	94.95	93.2

## Data Availability

No data were used to support this study.
